The article "Levosimendan Postconditioning Attenuates Cardiomyocyte Apoptosis after Myocardial Infarction" was retracted in 2023. Reasons: signs of a paper mill; suspected computer-generated content; unreliable results or conclusions; concerns about the data.

# Levosimendan Postconditioning Attenuates Cardiomyocyte Apoptosis after Myocardial Infarction

**DOI:** 10.1155/2022/2988756

**Published:** 2022-01-29

**Authors:** Ying Xie, Zhengjiang Xing, Jie Wei, Xiaolin Sun, Bin Zhao, Yan Chen, Yue Geng, Zheng Jia, Honglin Zou

**Affiliations:** Department of Cardiovascular Surgery, Yan'an Hospital Affiliated to Kunming Medical University, No. 245,Renmin East Road, Kunming, Yunnan Province 650051, China

## Abstract

**Background:**

Levosimendan preconditioning has been shown to attenuate myocardial apoptosis in animal models. However, protective effects of levosimendan postconditioning against myocardial apoptosis following myocardial infarction (MI) have not been evaluated. Therefore, we investigated the effects of levosimendan postconditioning on myocardial apoptosis in MI rat models.

**Methods:**

In an anoxia/reoxygenation (A/R) model, H9c2 cells were pretreated with or without levosimendan postconditioning after which their apoptosis rates were assessed by flow cytometry, RT-qPCR, and western blot analyses. Then, postconditioning was performed with or without levosimendan in MI rat models. Myocardiocyte apoptosis was evaluated by echocardiography, TTC staining, TUNEL staining, immunohistochemical staining, RT-qPCR, and western blot analysis.

**Results:**

Levosimendan postconditioning inhibited H9c2 cell apoptosis in A/R models by elevating Bcl-2 while suppressing Caspase-3 and Bax at both mRNA and protein levels. Moreover, it improved cardiac functions and reduced the left ventricle infarction area in MI rat models. Compared to the MI control group, cardiomyocyte apoptosis rates in the levosimendan postconditioning group were low. The reduced cardiomyocyte apoptosis rates were associated with downregulation of Bax and Caspase-3 as well as with upregulation of Bcl-2 at mRNA and protein levels.

**Conclusions:**

Levosimendan postconditioning of MI rat models protected against cardiomyocyte apoptosis, implying that it is a potential strategy for preventing cardiomyocyte apoptosis in the treatment of cardiac dysfunction following MI.

## 1. Introduction

Acute or chronic myocardial infarction is caused by myocardial cell ischemia following coronary artery obstruction, resulting in secondary myocardial cell necrosis [1]. Globally, myocardial infarction is associated with high death rates and significantly high treatment expenses [2, 3]. Myocardial infarction is a serious type of coronary heart disease, which is caused by acute or chronic myocardial ischemia after coronary artery system lumen or obstruction due to various reasons. Furthermore, myocardial necrosis occurs, which can lead to heart rupture, ventricular septal perforation, papillary muscle rupture, cardiogenic shock, heart failure, and even death. Therefore, the diagnosis of MI, device and drug treatment, and prevention as well as mechanism research on how to improve the function of cardiomyocyte are becoming the focus of research. It is a great significance for improving the heart function and survival rate of patients with MI [1, 4].

Levosimendan, a novel calcium sensitizer, has various pharmacological cardiovascular benefits, including positive inotropic with energy-saving cardiotonic effects, anti-inflammatory effects, and antiapoptotic effects [5, 6]. During open-heart surgery, levosimendan has been successfully used to treat preoperative and perioperative cardiac failure [7, 8]. Levosimendan preconditioning prevented myocardial ischemic damage and inhibited cardiomyocyte apoptosis in ischemia-reperfusion (I/R) models [9–13]. Clinically, in addition to ischemia-reperfusion injury, a significantly high number of patients present with myocardial infarction (MI) due to prolonged acute coronary artery occlusion. MI is associated with cardiomyocyte apoptosis, which is characterized by an irreversible loss of functioning cardiomyocytes, a reduction in coronary flow reserves, and cardiac dysfunctions [14]. In normal treatment, applications of levosimendan before acute myocardial infarction may be restricted [15]. Ischemic postconditioning has been shown to significantly reduce infarct sizes while exerting cardioprotective effects [16–19]. Therefore, MI patients may benefit from alternative therapeutic strategies including postconditioning to rescue ischemic myocardium and improve their surgical or survival outcomes. Recent studies have proposed levosimendan postconditioning treatment for MI. However, it has not been established whether levosimendan exerts protective effects against cardiomyocyte apoptosis following MI.

Levosimendan has been used well in clinical practice. To elucidate on the therapeutic effects of levosimendan postconditioning following MI, we investigated its antiapoptotic effects in *in vitro* anoxia-reoxygenation (A/R) models. Then, we established *in vivo* acute myocardial infarction (AMI) models to observe the effect of levosimendan on cardiomyocyte after MI. Thus, we will clarify a point to determine whether this treatment has protective effects against cardiomyocyte apoptosis following MI. This effect has a positive significance for clarifying the relevant mechanism of cardiomyocyte apoptosis.

## 2. Materials and Methods

### 2.1. Establishment of *In Vitro* H9c2 Cell Anoxia-Reoxygenation (A/R) Models

H9c2 cells were cultured in high-glucose Dulbecco's modified Eagle medium (DMEM) and presaturated for 1 h with 95% N_2_/5% CO_2_. To ensure (PO_2_) ≤ 4.0 kPa, O_2_ partial pressure was measured using a blood gas analyzer. Additionally, a reoxygenation medium was prepared and presaturated for 1 h with 95% O_2_/5% CO_2_ to maintain PO_2_ = 20.9 kPa.

The H9c2 cells (Shanghai Institute for Biological Sciences) were cultured in the anoxic media for 3 h and centrifuged. Then, anoxic H9c2 cells were placed in reoxygenation media for 2 h after which the cell suspension was centrifuged to obtain the cells. The anoxic/reoxygenated H9c2 cells were divided into two groups: A/R and the A/R + levosimendan (A/R + Levo) groups. Cells in the A/R group were cultured in normal media, while those in the A/R + Levo group were cultured in normal media supplemented with 0.3 µmol/L levosimendan (QILU Pharmaceutical, China). Additionally, control group cells without A/R were cultured in normal media. After 24 h, H9c2 cells from each group were digested, centrifuged, harvested, and used in subsequent experiments.

### 2.2. Flow Cytometry

An FITC Annexin V Apoptosis Detection Kit (BD, USA) was used to assay apoptotic H9c2 cells. In each fluorescence-activated cell sorting (FACS) tube, 100 *μ*l of cell suspension (1.0 × 10^6^ cells), 100 *μ*l of staining buffer, and 5 *μ*l of annexin V and propidium iodide were added, after which the samples were incubated as instructed by the manufacturer. Apoptotic cells were evaluated by a FACSCanto II flow cytometer with the FACSDiva 6.1.2 software (BD, USA) used for data analysis.

### 2.3. RT-qPCR

Total RNA was extracted from H9c2 cells using the TRIzol reagent (Invitrogen, USA), while the All-in-One™ First-Strand cDNA Synthesis Kit (GeneCopoeia, USA) was used for first-strand cDNA synthesis as instructed by the manufacturers. FastStart Universal SYBR Green Master (Roche, Germany) and the PikoReal 96-well system (Thermo Fisher, USA) were used for RT-qPCR analyses, which were performed in three independent experiments. Primers were designed using the Primer 5 software (Premier Biosoft International, Canada), with 5-CTCTCGTCGCTACCGTCGC-3 and 5-TCCCCCAGTTCACCCCATC-3 for Bcl2, 5-GGAACGAACGGACCTGTGGA-3 and 5-CGGGTGCGGTAGAGTAAGCA-3 for Caspase 3, and 5-CCGGCGAATTGGAGATGA-3 and 5-AGCGAGGCGGTGAGGACT-3 for Bax (all primers were synthesized by Sangon Biotech, China). The amount of each RNA sample was normalized to that of rat glyceraldehyde-3-phosphate dehydrogenase (GAPDH), the internal control.

### 2.4. Western Blotting

Caspase-3, Bax, and Bcl-2 were extracted from H9c2 cells and their expressions analyzed. After H9c2 cell lysis, protein concentrations were determined using a BCA protein assay kit (Beyotime, China). Protein samples (40 *μ*g) were loaded onto polyacrylamide gels, electrophoresed, and transferred onto nitrocellulose membranes. Nonspecific binding sites were blocked for 1 h using 5% nonfat dry milk. The blots were probed with Bax (1 : 5000 dilution, Abcam, UK), Caspase-3 (1 : 2000 dilution, Abcam, UK), and Bcl-2 (1 : 1000 dilution, Abcam, UK) antibodies. Goat-anti-rabbit IgG (1 : 5000 dilution, Millipore, USA) and goat anti-mouse IgG (1 : 5000 dilution, Millipore, USA) were used as secondary antibodies. The membranes were incubated 3–5 seconds with the enhanced chemiluminescence (ECL) detection reagent (Millipore, USA). The *β*-actin antibody (1 : 1000 dilution, Sigma-Aldrich, USA) was used as the internal standard. Protein bands were analyzed using the ImageJ software, with their concentrations being estimated relative to those of *β*-actin.

### 2.5. *In Vivo* Assays

Male Sprague-Dawley (SD) rats (160–200 g) were purchased from Kunming Medical University (Kunming, China). This study was approved by the Ethical Committee of Kunming Medical University and all animal procedures were performed in accordance with the National Institute of Health (NIH Publication No. 85–23, revised 2011) Guide for the Care and Use of Laboratory Animals. Rats were randomized into three groups: sham-operated group (sham group), MI group, and levosimendan postconditioning group (MI + Levo group).

Rats were anesthetized with intraperitoneally administered sodium pentobarbital (30 mg/kg), intubated, and ventilated during operation. The heart was exposed via left lateral thoracotomy and pericardiectomy. Then, using a 6.0 Prolene suture, the left anterior descending branch of the coronary artery was identified and gently ligated. Sham group rats were subjected to the same procedures, apart from ligation of the left anterior descending branch of the coronary artery. Successful MI was confirmed by observing myocardium color change from red to pale. Immediately following MI, rats in the MI + Levo group were intravenously infused with levosimendan (1.2 *μ*g/kg/min for 10 min followed by 0.2 *μ*g/kg/min for 1 h), while rats in the sham and MI groups were administered with equal amounts of 5% glucose solution.

### 2.6. Echocardiography

Transthoracic echocardiographic tests were performed on 7-day-old anesthetized rats using a GE VIVID E9 system equipped with a 10.0 MHZ probe. Left ventricle ejection fraction (LVEF), left ventricle end-diastolic diameter (LVEDd), and fractional shortening (FS) were obtained.

### 2.7. Tetrazolium Chloride (TTC) Staining

Following MI, all rats were sacrificed on the 7th day. Hearts were rapidly removed, washed, and placed in ice for 30 min at −20°C. Myocardial tissues from the left ventricle were sliced into 2 mm sections, which were then placed in 24-well plates. TTC was added to the wells, and the sections were incubated at 37°C for 30 min, followed by rinsing. Infarct areas in the left ventricle were marked and quantified using the Image-Pro Plus 6.0 software. The percentage of infarct area (%) = (*S*_*w*_/*S*_e_) × 100%, where *S*_*w*_ is the infarct area (white) and *S*_e_ is the entire cross-sectional area in the same layer.

### 2.8. Terminal Transferase-Mediated dUTP Nick End Labeling (TUNEL) Staining

Myocardial tissue samples were harvested from the left ventricle and fixed overnight in neutral buffered formalin. Then, they were dehydrated, cleared, paraffin-embedded, and sliced into 5 *μ*m sections for apoptosis analysis. Cardiomyocyte apoptosis was detected using the TUNEL assay kit (Roche, Germany). Nuclei of apoptotic cells were stained brown, while the nuclei of normal cells were stained blue. Moreover, morphological characteristics of apoptotic cells, including karyopyknosis, nuclear fragmentation, and karyolysis, were evaluated. Ten randomly selected high-powered fields (200× magnification) were examined in each section. Apoptotic rates (%) = (the number of apoptotic cells/total number of cells) ^*∗*^ 100.

### 2.9. RT-qPCR

Total RNA was extracted from frozen myocardial tissue samples using the TRIzol reagent (Invitrogen, USA), as instructed by the manufacturer. The rest of the procedures were similar to those used in RT-qPCR of H9c2 cells.

### 2.10. Western Blotting

Protein levels of Caspase-3, Bax, and Bcl-2 were evaluated using total protein extracted from myocardial tissue samples. The rest of the procedures were similar to those of western blot analysis as performed for H9c2 cells.

### 2.11. Immunohistochemical Staining

Paraffin-embedded sections were dewaxed and rehydrated, after which antigen retrieval was performed. To inactivate endogenous enzymes, sections were incubated with 3% H_2_O_2_ in deionized water at 37°C for 10 min. Then, they were incubated at 4°C overnight in the presence of anti-Bax (1 : 100 dilution, Abcam, UK), anti-Caspase-3 (1 : 100 dilution, Abcam, UK), and anti-Bcl-2 (1 : 100 dilution, Abcam, UK) primary antibodies. A biotin-labeled secondary antibody (ZsBio, China) was added, followed by incubation at 37°C for 40 min. Then, sections were stained with diaminobenzidine (DAB) for 5 min, counterstained with hematoxylin for 5 min, dehydrated, hyalinized, and sealed with neutral balsam. To detect brown cytoplasmic granules, sections were observed by light microscopy (Zeiss, Germany) connected to an Advanced 310 Image Processing system (Motic, Canada), to obtain the images.

### 2.12. Statistical Analysis

The SPSS 13.0 statistical software (IBM, USA) was used for all statistical analyses. Data are presented as mean ± SD. Between-group differences were assessed by the paired Student's *t*-test. *p* ≤ 0.05 was considered statistically significant.

## 3. Results

Levosimendan postconditioning inhibited H9c2 cell apoptosis in A/R models by elevating Bcl-2 and suppressing Caspase-3 as well as Bax expressions at the mRNA and protein levels.

Flow cytometry was performed to investigate apoptosis levels in each group of H9c2 A/R cell models (Figures 1(a) and 1(b) and Table 1). The A/R + Levo group exhibited a significantly low rate of apoptotic cells, compared to the A/R group (A/R + Levo 12.14 ± 0.94 versus A/R 21.41 ± 0.51, *p* < 0.05). To establish the apoptotic factors involved in the effects of levosimendan postconditioning in A/R H9c2 cell models, RT-qPCR (Figure 1(c) and Table 2) and western blotting (Figures 1(d) and 1(e) and Table 3) were performed to determine mRNA and protein levels of Caspase-3, Bax, and Bcl-2. Compared to the A/R group, the A/R + Levo group exhibited significantly suppressed Caspase-3 (A/R + Levo 1.17 ± 0.09 versus A/R 2.06 ± 0.13, *p* < 0.05) and Bax (A/R + Levo 1.91 ± 0.03 versus A/R 5.67 ± 0.34, *p* < 0.05) expressions at the mRNA levels, while Bcl-2 mRNA levels were significantly elevated (A/R + Levo 0.76 ± 0.004 versus A/R 0.32 ± 0.006, *p* < 0.05) (Figure 1(c) and Table 2, *p* < 0.05). Additionally, as shown in Figures 1(d) and 1(e), Bcl-2 protein levels were significantly upregulated (A/R + Levo 0.76 ± 0.06 versus A/R 0.63 ± 0.03, *p* < 0.05), while Caspase-3 (A/R + Levo 0.12 ± 0.02 versus A/R 0.26 ± 0.04, *p* < 0.05) and Bax (A/R + Levo 0.40 ± 0.06 versus A/R 0.81 ± 0.06, *p* < 0.05) protein levels were markedly downregulated in the A/R + Levo group, compared to the A/R group (Figures 1(d) and 1(e) and Table 3, *p* < 0.05). Compared to the control group, in the A/R + Levo group, Bcl-2 protein levels were suppressed (A/R + Levo 0.76 ± 0.06 versus control 0.98 ± 0.12, *p* > 0.05), while Caspase-3 (A/R + Levo 0.12 ± 0.02 versus control 0.13 ± 0.04, *p* > 0.05) and Bax (A/R + Levo 0.40 ± 0.06 versus control 0.34 ± 0.04, *p* > 0.05) protein levels were elevated. However, differences in expression levels between the control and A/R groups were not significant (Figure 1(e) and Table 3, *p* > 0.05).

### 3.1. Levosimendan Postconditioning Improved Cardiac Functions in MI Models

Echocardiographic measurements revealed that, on the 7th day after MI, rats receiving levosimendan postconditioning exhibited improved cardiac functions, compared to the MI group. Additionally, they exhibited significantly elevated LVEF and FS (Table 4, *p* < 0.05). As indicated by the significantly reduced LVEF as well as FS and elevated LVEDd, cardiac functions of the MI group were markedly decreased, compared to the sham group (Table 4, *p* < 0.05).

Levosimendan postconditioning attenuated myocardial injury and protected the myocardium against MI-induced cardiomyocyte apoptosis by elevating mRNA and protein levels of Bcl-2 while suppressing those of Caspase-3 and Bax. Of the thirty rats, MI was successfully established in 21 rats (70% success rate). The remaining 9 rats died due to anesthetic overdose, cardiac rupture, or other causes.

As shown in Figure 2(a), TTC staining revealed reduced areas of left ventricle infarctions in MI + Levo and MI groups (Figure 2(a)). The MI + Levo group had a lower percentage of infarct area, compared to the MI group (MI + Levo 18.03 ± 0.47 versus MI 20.58 ± 1.14, *p* < 0.05, Figure 2(b) and Table 5). TUNEL staining was performed to assess cardiomyocyte apoptosis following MI (Figures 2(a) and 2(c)). Compared to the control group, the MI and MI + Levo groups exhibited significantly more TUNEL-positive cell nuclei (brown) (Figure 2(a)). Interestingly, following MI, the MI + Levo group exhibited a lower percentage of apoptotic cardiomyocytes (brown), compared to the MI group (MI + Levo 0.15 ± 0.01 versus MI 0.21 ± 0.02, *p* < 0.05, Figure 2(c) and Table 6). RT-qPCR analysis revealed elevated Bcl-2 mRNA levels (MI + Levo 0.50 ± 0.08 versus MI 0.23 ± 0.07, *p* < 0.05) as well as significantly suppressed Caspase-3 (MI + Levo 2.84 ± 0.63 versus MI 5.73 ± 0.45, *p* < 0.05) and Bax (MI + Levo 7.91 ± 0.03 versus MI 15.67 ± 0.08, *p* < 0.05) mRNA levels in the MI + Levo group, compared to the MI group following MI (Figure 2(d) and Table 7). Western blotting analysis of myocardial tissues from each group revealed that, compared to the MI group, MI + Levo group had significantly suppressed Caspase-3 (MI + Levo 0.28 ± 0.02 versus MI 0.46 ± 0.04, *p* < 0.05) and Bax (MI + Levo 0.76 ± 0.06 versus MI 1.13 ± 0.16, *p* < 0.05) protein levels as well as elevated Bcl-2 protein levels (MI + Levo 0.87 ± 0.08 versus MI 0.69 ± 0.05, *p* < 0.05) (Figures 2(e) and 2(f) and Table 8). The immunohistochemical staining results for Caspase-3, Bax, and Bcl-2 were consistent with RT-qPCR and western blot analysis results (Figure 2(a)).

## 4. Discussion

Levosimendan preconditioning has been shown to protect cardiomyocytes against apoptosis [9–13]. Moreover, it exerted comparable antiapoptotic effects in organs such as the liver, lungs, and kidneys [20–24]. Even though recent studies have reported that pharmacological postconditioning is a potential method for preventing cardiac injury [25, 26], studies on levosimendan postconditioning are few, compared to those on levosimendan preconditioning. Generally, levosimendan is used in cases of appropriate clinical indications, such as definitive MI [5, 7, 8]. Based on findings from basic research and clinical practice, a hypothesis regarding the influence of levosimendan postconditioning on MI-induced myocardial apoptosis has been proposed. However, mechanisms of this levosimendan-conferred cardioprotection remain unclear. In this study, an *in vitro* A/R model, which is a suitable model for cell oxygen deprivation, was used [27, 28]. In A/R cell models, levosimendan postconditioning reduced the number of apoptotic H9c2 cells, compared to the control group. It is providing stronger and more direct evidence of levosimendan protective effects against reperfusion injury in clinical application.

It has been reported that one of the apoptotic pathways is tightly regulated by proteins from the B-cell lymphoma-2 (Bcl-2) family, such as Bcl-2, which have the ability to prolong cell survival by inhibiting apoptosis [29]. On the other hand, Bax, a member of the Bcl-2 family, promotes cell apoptosis [30]. Caspase-3, a member of the cysteine protease family, is a key apoptotic mediator and has the ability to cause cell death, as evidenced by the presence of cell lysates [31]. In A/R models in this study, levosimendan postconditioning enhanced Bcl-2 mRNA and protein levels while suppressing those of Caspase-3 and Bax. These findings could explain why levosimendan postconditioning attenuated H9c2 cell apoptosis. Moreover, levosimendan postconditioning exerted protective effects on H9c2 A/R cells.

Based on findings from *in vitro* experiments, we hypothesized that levosimendan can suppress myocardial apoptosis *in vivo* following MI. In MI rat models, compared to control treatment, levosimendan postconditioning after MI significantly reduced the number of apoptotic cardiomyocytes. Notably, it upregulated mRNA and protein levels of Bcl-2 while suppressing those of Caspase-3 and Bax in MI rat models, compared to control group. Histologically, levosimendan postconditioning was associated with a reduced left ventricular infarct area, compared to control treatment. Additionally, it partially improved cardiac functions following MI on the 7th day. Therefore, a reduction in the number of apoptotic cardiomyocytes and significant downregulation of proapoptotic protein levels following levosimendan postconditioning are beneficial factors in reducing the left ventricular infarct area and partially improving cardiac functions. Although this finding suggested that the therapeutic effect observed in our study was insufficient to completely reverse the damage caused by MI, our findings indicated a protective effect of levosimendan postconditioning against myocardial apoptosis. In other words, while some of the MI-induced apoptosis or necrosis in cardiomyocytes was irreversible, our findings revealed that levosimendan postconditioning can attenuate cardiomyocyte apoptosis and improve cardiac functions. Since the number of viable cardiomyocytes is critical for cardiac function improvements, levosimendan postconditioning, which exerts cardioprotective effects by inhibiting cardiomyocyte apoptosis following MI, may improve patient prognoses, thereby providing alternative strategies for interventions or surgical treatment.

## 5. Conclusions

Levosimendan inhibited apoptosis in H9c2 A/R cell models. Besides, *in vivo,* levosimendan postconditioning of MI rat models conferred cardioprotection by inhibiting cardiomyocyte apoptosis and improving cardiac functions.

## Figures and Tables

**Figure 1:** (a, b) Apoptosis of H9c2 cells in each group 24 h after A/R induction, as determined by flow cytometry (*n* = 5). (c) mRNA expressions of Caspase-3, Bax, and Bcl-2 in H9c2 cells in each group 24 h after A/R induction, as determined by RT-qPCR (*n* = 5). (d, e) Representative western blot images and quantitative analyses of Caspase-3, Bax, and Bcl-2 protein levels in H9c2 cells in each group 24 h after A/R induction (*n* = 5). A/R: anoxia-reoxygenation; Levo: levosimendan. #*p* < 0.05, A/R + Levo group versus A/R group; △*p* < 0.05, A/R + Levo group versus control group; ^*∗*^*p* < 0.05, A/R group versus control group.

**Figure 2:** (a, b) The left ventricular infarct area was detected by TTC staining in each group 7 days after MI model establishment (*n* = 3). (a, c) Representative TUNEL staining analysis of cardiomyocyte apoptosis in rats from each group 7 days after MI model establishment (*n* = 4). Normal cell nuclei are stained blue, while apoptotic cell nuclei are stained brown (magnification: × 200). (a) Immunohistochemical staining of Caspase-3, Bax, and Bcl-2 in rats from each group 7 days after MI model establishment (*n* = 4). Normal and apoptotic cell nuclei are stained blue and brown, respectively (magnification: × 100). (d) Caspase-3, Bax, and Bcl-2 mRNA levels in rats of each group 7 days after MI model establishment, as determined by qRT-PCR analysis (*n* = 4). (e, f) Representative western blot images and quantitative analyses of Caspase-3, Bax, and Bcl-2 protein levels in rats from each group 7 days after MI model establishment (*n* = 4). MI: myocardial infarction; Levo: levosimendan; ^#^*p* < 0.05, MI + Levo group versus MI group; ^Δ^*p* < 0.05, MI + Levo group versus control group; ^*∗*^*p* < 0.05, MI group versus control group.

**Table 1:** Apoptosis rates of H9c2 cells in each group 24 h after A/R induction.

	Control	A/R	A/R + Levo
Apoptosis (%)	7.58 ± 0.92	21.41 ± 0.51^*∗*^	12.14 ± 0.94^#△^

Data are presented as mean ± SD for *n* = 5. A/R: anoxia-reoxygenation; Levo: levosimendan. ^#^*p* < 0.05, A/R + Levo group versus A/R group; ^Δ^*p* < 0.05, A/R + Levo group versus control group; ^*∗*^*p* < 0.05, A/R group versus control group.

**Table 2:** mRNA expressions of Caspase-3, Bax, and Bcl-2 in H9c2 cells of each group 24 h after A/R induction.

	Control	A/R	A/R + Levo
Caspase-3	1	2.06 ± 0.13^*∗*^	1.17 ± 0.09^#^
Bcl-2	1	0.32 ± 0.006^*∗*^	0.76 ± 0.004^#^
Bax	1	5.67 ± 0.34^*∗*^	1.91 ± 0.03^#△^

Data are presented as mean ± SD for *n* = 5. A/R: anoxia-reoxygenation; Levo: levosimendan. ^#^*p* < 0.05, A/R + Levo group versus A/R group; ^Δ^*p* < 0.05, A/R + Levo group versus control group; ^*∗*^*p* < 0.05, A/R group versus control group.

**Table 3:** Protein levels of Caspase-3, Bax, and Bcl-2 in H9c2 cells of each group 24 h after A/R induction.

	Control	A/R	A/R + Levo
Caspase-3/*β*-actin	0.13 ± 0.04	0.26 ± 0.04^*∗*^	0.12 ± 0.02^#^
Bax/*β*-actin	0.34 ± 0.04	0.81 ± 0.06^*∗*^	0.40 ± 0.06^#^
Bcl-2/*β*-actin	0.98 ± 0.12	0.63 ± 0.03^*∗*^	0.76 ± 0.06^#^

Data are presented as mean ± SD for *n* = 5. A/R: anoxia-reoxygenation; Levo: levosimendan. ^#^*p* < 0.05, A/R + Levo group versus A/R group; ^Δ^*p* < 0.05, A/R + Levo group versus control group; ^*∗*^*p* < 0.05, A/R group versus control group.

**Table 4:** Parameters of cardiac functions in rats from each group 7 days after MI model establishment.

	Sham	MI	MI + Levo
LVEF (%)	76.99 ± 3.00	49.85 ± 2.65^*∗*^	57.25 ± 3.80^#△^
FS (%)	50.11 ± 3.24	42.15 ± 2.16^*∗*^	46.43 ± 2.93^#△^
LVEDd (mm)	4.90 ± 0.19	7.69 ± 0.21^*∗*^	6.68 ± 0.19^△^

Data are presented as mean ± SD for *n* = 7. LVEF: left ventricular ejection fraction; FS: fractional shortening; LVEDd: left ventricular end-diastolic diameter; MI: myocardial infarction; Levo: levosimendan; ^#^*p* < 0.05, MI + Levo group versus MI group; ^Δ^*p* < 0.05, MI + Levo group versus control group; ^*∗*^*p* < 0.05, MI group versus control group.

**Table 5:** Percentages of infarction areas in rats from each group 7 days after MI model establishment.

	Sham	MI	MI + Levo
The percentage of infarction area	0.00 ± 0.00	20.58 ± 1.14^*∗*^	18.03 ± 0.47^#△^

Data are presented as mean ± SD for *n* = 3. MI: myocardial infarction; Levo: levosimendan; ^#^*p* < 0.05, MI + Levo group versus MI group; ^Δ^*p* < 0.05, MI + Levo group versus control group; ^*∗*^*p* < 0.05, MI group versus control group.

**Table 6:** Apoptotic cardiomyocytes in rats from each group 7 days after MI model establishment.

	Sham	MI	MI + Levo
Apoptotic cells	0.03 ± 0.01	0.21 ± 0.02^*∗*^	0.15 ± 0.01^#△^

Data are presented as mean ± SD for *n* = 4. MI: myocardial infarction; Levo: levosimendan; ^#^*p* < 0.05 MI + Levo group versus MI group; ^Δ^*p* < 0.05, MI + Levo group versus control group; ^*∗*^*p* < 0.05, MI group versus control group.

**Table 7:** mRNA levels of Caspase-3, Bax, and Bcl-2 in rats from each group 7 days after MI model establishment.

	Sham	MI	MI + Levo
Caspase-3	1	5.73 ± 0.45^*∗*^	2.84 ± 0.63^#△^
Bcl-2	1	0.23 ± 0.07^*∗*^	0.50 ± 0.08^#△^
Bax	1	15.67 ± 0.08^*∗*^	7.91 ± 0.03^#△^

Data are presented as mean ± SD for *n* = 4. MI: myocardial infarction; Levo: levosimendan; ^#^*p* < 0.05, MI + Levo group versus MI group; ^Δ^*p* < 0.05, MI + Levo group versus control group; ^*∗*^*p* < 0.05, MI group versus control group.

**Table 8:** Protein levels of Caspase-3, Bax, and Bcl-2 in rats from each group 7 days after MI model establishment.

	Sham	MI	MI + Levo
Caspase-3/*β*-actin	0.21 ± 0.02	0.46 ± 0.04^*∗*^	0.28 ± 0.02^#^
Bax/*β*-actin	0.58 ± 0.03	1.13 ± 0.16^*∗*^	0.76 ± 0.06^#^
Bcl-2/*β*-actin	1.24 ± 0.06	0.69 ± 0.05^*∗*^	0.87 ± 0.08^#△^

Data are presented as mean ± SD for *n* = 4. MI: myocardial infarction; Levo: levosimendan; ^#^*p* < 0.05, MI + Levo group versus MI group; ^Δ^*p* < 0.05, MI + Levo group versus control group; ^*∗*^*p* < 0.05, MI group versus control group.

## Data Availability

The simulation experiment data used to support the findings of this study are available from the corresponding author upon request.
